The article "Prick-by-Prick Test with Pasteurised Cow's Milk: A Valuable Tool in Paediatric Practice" was published in 2022. Journal: Biomed Res Int.

# Prick-by-Prick Test with Pasteurised Cow's Milk: A Valuable Tool in Paediatric Practice

**DOI:** 10.1155/2022/9738654

**Published:** 2022-09-07

**Authors:** Ieva Adomaite, Neringa Stirbiene, Vilma Marciukaitiene, Laura Akuleviciute, Romualdas Gurevicius, Sigita Petraitiene, Odilija Rudzeviciene

**Affiliations:** ^1^Clinic of Children's Diseases, Institute of Clinical Medicine, Faculty of Medicine, Vilnius University, Vilnius, Lithuania; ^2^Centre of Paediatrics, Vilnius University Hospital Santaros Clinics, Vilnius, Lithuania; ^3^Centre of Health Information, Institute of Hygiene, Vilnius, Lithuania

## Abstract

**Background:**

This study assessed the utility of a prick-by-prick test with pasteurised cow's milk in predicting a pasteurised cow's milk allergy (CMA) diagnosis.

**Methods:**

This was a retrospective study of 86 paediatric patients who had undergone open pasteurised cow's milk oral food challenges (OFCs). We evaluated the diagnostic performance of a prick-by-prick test with pasteurised cow's milk in predicting a positive OFC result. We calculated the threshold values representing high test specificity and predictive probability in children aged ≤24 and >24 months.

**Results:**

A prick-by-prick test with pasteurised cow's milk was a good classifier of a positive cow's milk OFC outcome. The mean prick − by − prick test wheal diameter ≥ 3 mm yielded 100% sensitivity in both groups of children. Thresholds representing high test specificity and 95% predicted probability were 7 and 11 mm in children ≤ 24 months and 11 and 17 mm in children > 24 months of age, respectively.

**Conclusion:**

A prick-by-prick test with pasteurised cow's milk is valuable in paediatric practice when diagnostic thresholds are implemented.

## 1. Introduction

Cow's milk is one of the most common food allergens and an essential source of nutrients in infancy and early childhood [1, 2]. An accurate cow's milk allergy (CMA) diagnosis is essential to avoid allergic reactions in allergic individuals and prevent unnecessary dietary restrictions in those without allergies [3]. The double-blind placebo-controlled food challenge (DBPCFC) test is considered the “gold standard” of food allergy testing [4]. Nevertheless, due to its complexity, it is mainly used for research purposes and when an open oral food challenge (OFC) result is ambiguous [5]. Open OFCs are less demanding yet still time-consuming and require trained medical personnel. This makes the availability of DBPCFCs and OFCs limited.

Considering the growing number of allergic children and a specialist shortage [6, 7], children with suspected CMA are often managed by their primary care physician or paediatrician long before having access to an allergy specialist. This presents a demand for a convenient, rapid, and cost-effective method to confirm or reject a CMA diagnosis in a primary care setting.

Tests used to verify immunoglobulin E- (IgE-) mediated food sensitisation such as skin prick tests with commercial extracts are rapid and relatively inexpensive [8]; however, only standardised commercially available allergen extracts that have comparable antigenic compositions between different manufacturers should be used, and the potency of the allergen extract can deteriorate with time [8, 9]. Serum-specific IgE (sIgE) antibody test results can differ between various methods and require expertise to interpret the test results [9]. Measuring the level of serum food sIgE is helpful in diagnosing food allergy, especially when the threshold values above 95% predictive probability are implemented [10]. Nevertheless, both skin prick tests and food sIgE tests are not universally available to all primary care physicians and thresholds that establish the presence of sensitisation lack specificity to diagnose CMA [11].

A prick-by-prick (PBP) test performed with pasteurised cow's milk could be a possible solution to provide a CMA testing tool to most primary care physicians; however, appropriate quality and safety measures must be used, and threshold values that confirm or exclude CMA need to be employed to avoid misdiagnosis [9, 11]. The use of the prick-by-prick test is long-standing in CMA diagnosis, yet the threshold values indicative of a positive cow's milk OFC result in children of different ages have not been sufficiently explored. Therefore, we aimed to assess the utility of the PBP test with pasteurised cow's milk and define highly sensitive and specific threshold values in predicting a pasteurised CMA diagnosis in children.

## 2. Materials and Methods

### 2.1. Study Population

This was a retrospective medical record study of 86 paediatric patients with suspected or confirmed CMA. Controlled open OFCs were conducted at Vilnius University Hospital Santaros Clinics Centre of Paediatrics between 2011 and 2019. Two researchers analysed medical record data and OFC protocols. Data with ambiguous OFC results were not included. Patients were referred for an OFC because of a positive history of reactions or sensitisation to milk confirmed by a positive pasteurised cow's milk PBP test or elevated milk sIgE levels.

Children with vague reactions or sensitised but unexposed to milk were challenged to clarify the allergy status. When oral tolerance was suspected, repeated challenges were carried out in children with an established CMA. Prick-by-prick tests were performed in all children using pasteurised cow's milk containing 2.5% fat with single-head metal prick lancets by trained nurses per standard procedure [8]. Open OFCs were conducted using pasteurised cow's milk or cow's milk formula (for infants under 12 months); in addition, data of four children that failed heated milk challenges were included as they were considered to be allergic to pasteurised cow's milk (patient nos. 4, 8, 13, and 18 in Table 1). The challenges were performed with increasing doses given at 20-minute intervals, with a cumulative protein dose of 2.7 g in infants under 12 months and 4.4- 6.8 g in older children. An immediate reaction was considered positive when objective symptoms were noted during the challenge or within a two-hour observation period after the final challenge dose. Objective symptoms indicative of immediate reactions reported during the positive challenges were anaphylactic reaction (defined by the clinical criteria for diagnosing anaphylaxis) [12], skin symptoms (generalised erythema, macular or maculopapular rash, urticaria, and angioedema), rhinitis and conjunctivitis, gastrointestinal symptoms (vomiting and diarrhoea), respiratory symptoms (stridor, coughing, and wheezing), and cardiovascular symptoms. Immediate reactions were considered negative if no symptoms were observed for two hours after ingesting the age-appropriate amount of food. The Vilnius Regional Biomedical Research Ethics Committee provided ethical approval to perform this retrospective study, and the requirement for informed consent was waived.

### 2.2. Statistical Analysis

The discriminatory value of the PBP test to predict the OFC outcome was assessed by receiver-operating characteristic (ROC) analysis to determine the area under the curve (AUC). The threshold values representing high test specificity were determined from the ROC analysis. As proposed by Sampson, logistic regression was used to determine 95% predictive probability thresholds [10]. Two-by-two tables were used to compute the sensitivity and specificity values of the defined test thresholds. Positive and negative likelihood ratios and 95% confidence intervals were calculated using the MedCalc diagnostic test evaluation calculator [13]. Analyses were performed using SPSS for Windows (release 27.0.1; SPSS Inc., Chicago, IL, USA). *P* values of ≤0.05 were considered statistically significant.

## 3. Results

The medical records of 86 children who had undergone 98 OFCs were analysed. Most of the children were male 59 (68.6%). The median age of children at the time of the OFC was 23 months (1.9 years), ranging from 6 to 129 months (0.5 to 10.8 years). Fifty-two (53.1%) OFCs were performed in children aged ≤24 months and 46 (46.9%) in children >24 months of age. The demographic and clinical characteristics of the study population are shown in Table 2.

There were 18 (18.4%) positive OFCs in children aged 7 to 100 months (0.6 to 8.3 years). The most common symptoms observed during the positive OFCs were skin symptoms in 14 (77.8%) OFCs. Anaphylaxis developed in two positive OFCs (11.1%), and isolated respiratory symptoms were observed in two (11.1%) positive OFCs (Table 1).

The mean cow's milk PBP wheal diameters ranged from 0 to 22.5 mm (median 3 mm). The ROC analysis revealed that a PBP test with pasteurised cow's milk was a good classifier of a pasteurised cow's milk OFC outcome, with an AUC value of 0.94 in children ≤ 24 months of age (*P* < 0.001) and 0.86 in children > 24 months of age (*P* = 0.001) (Figure 1). The mean PBP test wheal diameter of ≥3 mm yielded 100% sensitivity in both groups of children. In children ≤ 24 months of age, the mean PBP test wheal diameter of 7 mm demonstrated a 97.7% specificity. The mean wheal size diameter predictive of a 95% positive oral challenge was 11 mm and was no more specific than the 7 mm threshold value (Table 3).

In children > 24 months of age, the mean PBP test wheal diameter of 11 mm demonstrated 94.4% specificity. The mean wheal size diameter predictive of a 95% positive oral challenge was 17 mm and demonstrated 100% specificity (Table 3).

## 4. Discussion

It is known that the generally suggested thresholds of commonly used allergy tests that establish the presence of food sensitisation are sensitive but lack specificity [11]; thus, a CMA diagnosis should not be made based solely on these threshold values. Despite its cost and possible risks, an OFC remains integral for making the definitive CMA diagnosis [4].

Nevertheless, with the number of allergic children increasing and the allergy specialist care becoming less readily available [2, 7], a convenient, rapid, and cost-effective method to confirm or reject a CMA diagnosis is required in a primary care setting. A prick-by-prick test with pasteurised cow's milk is a rapid, inexpensive, and universally available test that can be utilised in paediatric primary care if appropriate quality and safety measures are used and threshold values that confirm or exclude CMA are applied [9].

In our study, we found that a PBP test with pasteurised cow's milk has a good discriminatory power to predict a pasteurised cow's milk OFC outcome; the AUC value was 0.94 in children ≤ 24 months of age and 0.86 in children > 24 months of age. In a study by Verstege et al. (median patient age 22 months, ranging from 3 months to 14.5 years), the estimated AUC value was 0.82, Mauro et al. (mean patient age 3.6 ±2.9 years) reported a 0.87 value, and Onesimo et al. (median patient age 2.74 years, ranging from one month to 15 years) estimated the AUC value of 0.83 [14–16]. These studies did not calculate the different AUC values for separate age groups; therefore, they correspond more to our estimate for older children.

We found that the mean PBP test wheal diameter ≥ 3 mm yielded 100% sensitivity in both groups of children. The previously mentioned authors reported sensitivity ranging from 85% to 96.4% [14–16].

The mean PBP wheal diameter thresholds representing high test specificity and 95% predicted probability were 7 and 11 mm in children ≤ 24 months of age and 11 and 17 mm in children > 24 months of age, respectively. Similarly, Verstege et al. defined a mean fresh milk PBP 95% predictive threshold value of 9.7 mm in infants under one year of age and 15.7 mm in older children [14]. Other studies have defined 95% predicted probability threshold values ranging between 10 and 15 mm, although they did not stratify the threshold values by age [15, 17, 18].

A systematic review has summarised the results of multiple studies analysing sensitisation test accuracy in diagnosing milk allergy and proposed predictive test thresholds for accurately suspecting a pasteurised CMA [11]. The authors noted significant variation between the study results, which was explained by differences in the composition of the study populations, diagnostic and OFC methods, and statistical approaches [11]. This review could not conclude a diagnostic cow's milk PBP test threshold value in children over two years, but a mean wheal diameter above 8 mm for pasteurised cow's milk PBP test in patients under two years of age was suggested as predictive for pasteurised CMA [11]. In contrast to this variability in published thresholds, our 7 mm threshold for children ≤ 24 months is comparable to the one indicated by this systematic review.

Our study shows that a PBP test with pasteurised cow's milk is very sensitive. When no strong anamnestic and clinical evidence of IgE-mediated food allergy is present, a mean pasteurised cow's milk PBP test wheal diameter of <3 mm is sufficient to exclude an IgE-mediated CMA.

We suggest using high specificity and predicted probability values as communication tools with cow's milk allergic patients and their parents. Ultimately, the decision to perform an OFC must be made with respect to their views and preferences. A high specificity value of 7 mm may be preferred as a decision point to withhold a pasteurised cow's milk OFC in children ≤ 24 months, as the high probability of positive OFC reactions may not be acceptable for some parents. Tolerance may develop spontaneously in a number of CMA patients; therefore, some may prefer a watchful waiting tactic in this age group [19]. Baked milk OFC could be suggested in these patients, as most cow's milk allergic children can tolerate baked milk and its inclusion in the patient's diet could accelerate the development of tolerance to pasteurised milk [20]. In children > 24 months, the decision to withhold a pasteurised cow's milk OFC based on the high specificity or predicted probability values should be used with consideration, especially in older children, as children over four years of age with persistent CMA may benefit from oral allergen immunotherapy [21]. Therefore, even a positive pasteurised cow's milk OFC outcome could lead to an intervention instead of continuing food avoidance.

When high sensitivity and specificity thresholds are implemented, a fraction of patients remain in the “grey area,” where their sensitisation test values are not low enough to exclude the diagnosis of allergy and not high enough to be classified as allergic by the test. These patients will require an OFC for determining their allergy status, but even in this case, thresholds can be utilised to provide informed decision-making on the allergy management. If the decision to withhold a pasteurised cow's milk OFC is made, it should be periodically reevaluated alongside the sensitisation status of the patient.

## 5. Conclusion

In conclusion, a prick-by-prick test with pasteurised cow's milk is valuable in paediatric practice when age-appropriate diagnostic thresholds are implemented.

## Figures and Tables

**Figure 1:** Receiver-operating characteristic analysis showing the performance of pasteurised cow's milk prick-by-prick test in relation to the diagnosis of pasteurised cow's milk allergy in children aged ≤24 and >24 months.

**Table 1:** The characteristics of the patients with positive oral food challenge reactions.

Patient number	Patient age (months)	Form of milk used during the OFC	Mean cow's milk PBP wheal diameter (mm)	Cumulative protein dose reached (g)	Symptoms
1.	7	Infant formula	5.5	2.9	MP rash, diarrhoea
2.	12	Infant formula	7	0.2	MP rash
3.	12	Infant formula	9.5	2.9	MP rash
4.	19	Milk powder	9	4.4	Cough, wheezing
5.	20	Pasteurised	5.5	2.8	Diffuse erythema, conjunctivitis
6.	21	Pasteurised	6.5	6.8	MP rash
7.	22	Pasteurised	6.5	3.5	Urticaria, cough
8.	24	Milk powder	6	2.6	Skin erythema, diarrhoea, drowsiness
9.	25	Pasteurised	8	0.2	Anaphylaxis
10.	28	Pasteurised	7	1.8	Urticaria
11.	29	Pasteurised	6	0.4	Anaphylaxis
12.	31	Pasteurised	8	0.7	Urticaria
13.	31	Milk powder	4	2.6	Urticaria
14.	33	Pasteurised	9	6.8	Urticaria
15.	42	Pasteurised	9.5	0.2	MP rash
16.	48	Pasteurised	6	2.5	Diffuse erythema
17.	64	Pasteurised	6	6.8	Diffuse erythema, conjunctivitis
18.	100	Baked milk	22.5	4.4	Cough, wheezing

OFC: oral food challenge; PBP: prick-by-prick test; MP: maculopapular.

**Table 2:** Demographic and clinical characteristics of the study population.

Characteristic	*N* (%)
Patients	86 (100.0)
Male gender	59 (68.6)
Clinical history	
Atopic dermatitis	70 (81.4)
Asthma	12 (14.0)
Rhinitis	21 (24.4)
Parent reported food allergy symptoms	
Urticaria and/or angioedema	17 (19.8)
Anaphylaxis	10 (11.6)
Gastrointestinal symptoms	21 (24.4)
Family history of atopic diseases	30 (34.9)

**Table 3:** The diagnostic performance of standard thresholds representing a positive prick-by-prick test and optimal thresholds representing a high test specificity and predicted probability.

Patient age	≤24 months		>24 months	
Statistic	Value	95% CI	Value	95% CI
Area under the curve	0.94	0.88–1.00	0.86	0.75–0.97
*P* value	<0.001		0.001	
Positive PBP threshold	3 mm		3 mm	
Sensitivity (%)	100.0	63.1 to 100.0	100.0	69.2 to 100.0
Specificity (%)	68.2	52.4 to 81.4	50.0	32.9 to 67.1
LR+	3.1	2.0 to 4.8	2.0	1.4 to 2.8
LR-	0.0	-	0.0	-
High specificity PBP threshold	7 mm		11 mm	
Sensitivity (%)	37.5	8.5 to 75.5	10.0	0.3 to 44.5
Specificity (%)	97.7	88.0 to 99.9	94.4	81.3 to 99.3
LR+	16.5	2.0 to 139.4	1.8	0.2 to 17.9
LR-	0.6	0.4 to 1.1	1.0	0.8 to 1.2
95% predicted probability PBP threshold	11 mm		17 mm	
Sensitivity (%)	0.0	0.0 to 36.9	10.0	0.3 to 44.5
Specificity (%)	97.7	88.0 to 99.9	100.0	90.3 to 100.0
LR+	0.0	-	0.0	-
LR-	1.0	1.0 to 1.1	0.9	0.7 to 1.1

PBP: prick-by-prick test; LR+: positive likelihood ratio; LR-: negative likelihood ratio.

## Data Availability

The data used to support the findings of this study are available from the corresponding author upon request.
